This article has been retracted.

# Establishment and Analysis of Hypoxia-Related Model in Oral Squamous Cell Carcinoma

**DOI:** 10.1155/2022/6602648

**Published:** 2022-04-07

**Authors:** Xingwei Lu, Xingguang Liu

**Affiliations:** ^1^Department of Oral and Maxillofacial Surgery, School and Hospital of Stomatology, Cheeloo College of Medicine, Shandong University & Shandong Key Laboratory of Oral Tissue Regeneration & Shandong Engineering Laboratory for Dental Materials and Oral Tissue Regeneration, Jinan, China; ^2^No. 1 Ctomatology Department, The Volgograd State Medical University Volgograd Regional Clinical Hospital Volgograd, Volgograd Oblast, Russia

## Abstract

Oral squamous cell carcinoma (OSCC) is one of the most common cancers in the world. Hypoxia is closely related to immunity in tumor microenvironment and also affects the prognosis of patients. However, there is still a lack of articles related to tumor hypoxia in oral squamous cell carcinoma. Therefore, we aimed to develop a hypoxia model for future application in patient prognosis analysis and immunotherapy. The transcriptome and survival information of OSCC were downloaded from GEO database. The Cox regression model of the lasso method was used to identify prognostic genes and develop gene characteristics based on hypoxia immunity. According to the median risk value, the patients were divided into high-risk group and low-risk group. Then, the estimated algorithm was used to estimate the relationship between hypoxia and immune status. At the same time, we evaluated the correlation and expression differences of immune-related genes between different risk groups. By using the lasso model, we identified two genes, including PFKP and SERPINE1, to construct gene signatures for risk stratification. We observed that both genes were highly expressed in the high-risk group, which was not conducive to the prognosis of the tumor. In addition, in the analysis of the degree of immune infiltration, we observed that there were differences in the content of a variety of immune cells between the two groups. It can be seen that there were great differences in the immune cells constituting the tumor microenvironment in oral squamous cell carcinoma. There remain significant differences in the expression levels of multitudinous immune-related genes. These immune-related genes include CCL chemokines, Chemokine (C-X-C motif) ligand (CXCL), CD antigens, HSP family, interferon family, and interleukin family. The hypoxia-immune-based gene signature represents a promising tool for risk stratification tool in oral squamous cell carcinoma cancer. It might serve as a prognostic classifier for clinical decision-making regarding individualized prognostication and treatment and follow-up scheduling.

## 1. Introduction

Squamous cell carcinoma is the major malignant tumor of oral mucosa and lips [1]. Its incidence is especially high in western countries [2]. As far as we know, the main risk factors of oral squamous cell carcinoma (OSCC) include human papillomavirus (HPV), tobacco, and alcohol [3]. HPV-positive OSCC and HPV-negative OSCC are two different squamous cell carcinomas [4]. There are many differences in geographical distribution and clinicopathological and biological characteristics [5]. In this study, our subjects were negative oropharyngeal squamous cell carcinoma.

Hypoxia is one of the signs of cancer and is common in various solid tumors and plays an important role in the occurrence and development of tumors. It is caused by insufficient oxygen supply, mainly due to the disorder and defect of tumor microcirculation. In recent years, more and more studies began to pay attention to the role of hypoxia in tumor development. Some studies have pointed out that microfibrillar-associated protein 5 (MFAP5) is highly expressed in a variety of cancers, and it is observed that the overexpression of mfap5 is related to lymph node metastasis and poor prognosis of head and neck squamous cell carcinoma (HNSCC) [6]. Subsequently, it is observed that the expression of MFAP5 increases significantly in HNSCC cell line when the cells are under hypoxia. MFAP5-overexpressed cell lines had significantly higher migration and invasion abilities. In addition, in vivo analysis showed that overexpression of MFAP5 could promote tumor lung metastasis. Experiments show that MFAP5 may promote this process by activating epithelial mesenchymal transformation (EMT) through Akt pathway [7]. In addition, studies have found that hypoxia-induced ZEB1 can promote the progression of cervical cancer through CCL8-dependent recruitment of tumor-associated macrophages [8].

In addition to hypoxia-mediated resistance to standard therapies, regulation of gene and protein expression, genetic instability, and malignant progression, hypoxia also plays a key role in anticancer immune response [9]. At present, the common treatment methods of oral cancer include surgery, radiotherapy, chemotherapy and anti-EGFR drugs [10]. Immunotherapy is gradually developing into mature treatment methods, such as anti-CTLA-4 treatment and anti-PD-L treatment [11]. Several papers have discussed new molecular markers, but there are few clinical trials on them [12]. At present, immunotherapy is a new treatment option for oral cancer. The purpose of our study was to establish a hypoxia-related model in OSCC to speculate the prognostic value for patients with OSCC.

## 2. Materials and methods

### 2.1. Extraction of Original Data and Hypoxia-Related Genes

The OSCC-associated RNA sequencing and clinical data GEO (gse41613) database were used in this study. We downloaded the names of all hypoxia-related genes from the GSEA website (https://www.gsea-msigdb.org/gsea/index.jsp). The hypoxia gene network was constructed using STRING database (http://string-db.org/cgi/input.pl). The 50 genes with the largest number of adjacent nodes were selected by *R* software for subsequent analysis.

### 2.2. Construction of Hypoxia Model and Prognostic Analysis

In order to establish the score of hypoxia, first, we performed univariate Cox regression analysis to explore prognostic genes. Subsequently, lasso regression analysis was performed to establish hypoxia-related scores. The formula for calculating hypoxia-related score was as follows: score = (coefficient of mRNA1 × expression of mRNA1) + (coefficient of mRNA2 × expression of mRNA2) + ⋯ + (coefficient of mRNAn × expression mRNAn). In addition, in order to study the correlation between hypoxia-related score and overall survival, we used the “survival” package for survival analysis. Patients were divided into high-risk group or low-risk group according to the median risk score. In order to further verify the hypoxia-related score, the receiver operating characteristic (ROC) curve was constructed to check the accuracy of prognosis. In this study, the pheatmap package in *R* was used to draw the heat map of gene expression.

Correlation between immune gene expression and immune infiltration and hypoxia risk CIBERSORT is used to calculate the ratios of immune cell types in low- and high-risk classes. In each sample, the number of all predicted immune cell type scores equals 1. The online platform (http://biocc.hrbmu.edu.cn/TIP/index.jsp) for tracking tumor immunophenotypes to screen for immune-related genes plays an important role in the control of this immune cell type. After screening for genes that play a key role in immune cell regulation, the ggplot2, ggpubr, and ggExtra packages in *R* were used to analyze the correlations between gene expression and the risk of hypoxia.

### 2.3. Gene Set Enrichment Analysis

We downloaded the HALLMARK gene set and gene symbols from the GSEA website (https://www.gsea-msigdb.org/gsea/index.jsp) to extract hypoxia-related genes. The entire transcriptome of all tumor samples was used for GSEA, and only gene sets with nominal *P*-values <0.05 were considered significant.

## 3. Results

### 3.1. Construction of Hypoxia-Related Model

After downloading the data of oral squamous cell carcinoma, we used the string website to construct the PPI between hypoxia-related genes (Figure 1(a)). By calculating the number of adjacent nodes of each protein, we determined the core gene. Subsequently, the top 50 core genes with the largest number of adjacent nodes were identified (Figure 1(b)). Then, we screened the genes related to prognosis using univariate Cox regression analysis (Figure 1(c)). Among the identified genes, ENO1, PFKFB3, PFKP, SDC2, SDC4, SERPINE1, and SLC2A3 were further revealed by multivariable Cox regression analysis (Figure 1(d)) and then used to construct the prognosis model. The two genes are PFKP and SERPINE1. We observed that these two genes coefficients were 2.350 and 1.795, respectively, indicating that these two genes are associated with a high risk of tumor malignancy.

### 3.2. Hypoxia Risk Score Shows Great Feasibility for Prognosis

The patients were divided into high-risk group and low-risk group according to the appeal method. Survival analysis showed that the long-term survival rate of high-risk group was significantly lower than that of low-risk group, and there was significant difference between the two groups (*P* < 0.05; Figure 2(a)). Receiver operating characteristic curve analysis showed that the accuracy of predicting 1-year, 3-year, and 5-year survival rates of patients in oral squamous cell carcinoma database was relatively high, and the area under all ROC curves was >0.8 (Figure 2(b)). This showed that the accuracy of survival estimation obtained from this model is high and meaningful. We used risk histogram to show the difference of survival status between the two databases. We observed that the proportion of surviving patients in the low-risk group was higher than that in the high-risk group. We observed that the survival rate in the low-risk group was 67%, while the survival rate in the high-risk group was only 27% (Figure 2(c)). We also analyzed the interaction between hypoxia-related genes in the model. Obviously, there was a positive correlation between the two genes (Figure 2(d)). Both genes were unfavorable to the prognosis of cancer. Therefore, we speculated that the two genes promote the development of cancer.

We observed that the survival time of the low-risk group was longer than that of the high-risk group. In addition, the number of deaths in the low-risk group decreased over time (Figure 3(a)). We further demonstrated the relationship between patient risk and survival using a risk curve, in which the risk scores of the two groups of patients were plotted (Figure 3(b)). Finally, we compared the expression levels of each gene contained in the model between the high-risk and low-risk groups using heatmap. Finally, we found that both genes were highly expressed in the high-risk group (Figure 3(c)).

### 3.3. Analysis between Hypoxia and Immune Infiltration

CIBERSORT method was used to analyze the infiltration of 22 immune cell subsets. We observed that there were rich differences in the infiltration of 11 immune cell subsets between high-risk and low-risk groups (Figure 4(a)). We observed that activated dendritic cells, eosinophils, M0 macrophases, resting NK cells, and neutrophils were highly expressed in the high-risk group. Naive B cells, M2 Macrophages, activated Mast cells, resting Mast cells, plasma cells, follicular helper T cells, and gamma delta T cells were highly expressed in the low-risk group (Figure 4(b)).

### 3.4. Expression of Immune-Related Genes in High- and Low-Risk Groups

Resorting to the online platform “track tumor immune phenotype” (http://biocc.hrbmu.edu.cn/TIP/index.jsp), we screened immune-associated genes and sought for those that are critical to regulate this immune cell type. We drew a heatmap to visualize the expression of these genes pertaining to hypoxia-associated genes in the high-risk and low-risk patient groups in the GEO database (Figure 5(a)). There remain significant differences in the expression levels of multitudinous immune-related genes (*P* < 0.05). These immune-related genes include CCL chemokines, Chemokine (C-X-C motif) ligand (CXCL), CD antigens, HSP family, interferon family, and interleukin family (Figures 5(b)–5(g)).

### 3.5. GSEA Identifies Hypoxia Signaling Pathways

Using GSEA software, we analyzed the enrichment pathways of hypoxia-related genes in high-risk and low-risk groups. Interestingly, we observed that the high-risk groups were enriched in the pathways related to hypoxia and tumor process, including glycolysis, angiogenesis, hypoxia, TGF beta signaling, mitotic spindle, TNFA signaling via NF-kB, and epithelial mesenchymal transition (Figure 6).

The low-risk group did not have this feature, and the enriched pathways were more concentrated in fat acid metabolism, bile acid metabolism, peroxisome, and KRAS signaling (Figure 7).

## 4. Discussion

Hypoxia is a common feature of malignant tumors. Hypoxia interacts with chemical resistance, radiation resistance, invasiveness, and angiogenesis. Therefore, more and more studies believe that tumor hypoxia is an effective target for the treatment of cancer [13].

In our research, we found that core genes (PFKP and SERPINE1) are closely related to the prognosis of patients. The progression and prevalence of cancer are highly correlated with glycolysis [14]. As one of the rate limiting enzymes of glycolysis, the abnormal expression of PFKP has been reported in different types of cancer [15–17].

Phosphofructokinase-1 (PFK-1) is an allosteric enzyme that determines the rate of glycolysis and regulates the oxidation of glucose in cell respiration [18]. PFKP is mainly an isomer existing in platelets, and it is also a subtype of Phosphofructose kinase-1 (PFK-1). PFK-1 is a rate controlling enzyme in glycolysis. It can catalyze the phosphorylation of fructose 6-phosphate (F6P) to fructose 1, 6-diphosphate (F1, 6BP) [19]. When HIF-1*α* were knocked down in mature brown adipocytes, a decrease in PFKP expression was observed in adipocytes, indicating that PFKP is one of the HIF-1 *α* targets [20]. A recent progress has revealed that KLF4 mediated PFKP regulation. KLF4 is a transcription factor that upregulates glycolytic metabolism by directly binding to the promoter region of PFKP gene [21]. PFKP plays an important role in glycolysis. The GSEA analysis of this study also observed that one of the enriched pathways in the high-risk group is glycolysis.

Serpine1 gene is one member of the serine protease inhibitor superfamily, which is the main regulator of plasminogen activator system (PAs) [22]. The SERPINE1 gene is located at 7q21.2-q22 and codifies for a single-chain glycoprotein of about 50 kDa [23]. In recent years, studies have begun to pay attention to the role of serpine1 in head and neck squamous cell carcinoma. Studies have shown that SERPINE1 and SMA expression could predict extracapsular spread and survival in oral squamous cell carcinoma [24]. It is speculated that serpine1 promotes tumor cell migration and invasion, which may be mediated by Akt phosphorylation and activation [25]. In addition, we also found that serpine1 interacted with LRP1 to promote the migration of tumor cells [26]. The above analysis showed that PFKP and SERPINE1 may play an important role in oral squamous cell carcinoma and may also be used as new predictive molecules of oral squamous cell carcinoma.

It is reported that tumor microenvironment components and immune system biomarkers are important for cancer detection and evaluation of prognosis and treatment response [27–29]. The examination of tumor microenvironment has important prognostic value and can supplement histopathology and molecular biomarkers to evaluate the patient's response to treatment. Therefore, we analyzed the immune infiltration components in oral squamous cell carcinoma. We found that there were significant differences in the composition of a large number of immune cells in cancer cells. The different immune microenvironment may be the reason for the different prognosis of high-risk and low-risk groups. After analyzing the relationship between immune-related genes and high-risk groups, we observed that a large number of immune-related genes were differentially expressed in high-risk groups. These genes need further analysis in the future, or they can become new checkpoint inhibitors. The molecular mechanisms related to the development and drug resistance of oral squamous cell carcinoma remain largely unknown.

It is particularly important to understand the new biomarkers related to oral squamous cell carcinoma for the judgment and treatment of tumor prognosis. The establishment of a new prognosis model is helpful to determine the specific targets of biotherapy and optimize treatment and patient care. In addition, in some cases, the pathogenesis of such tumors may be conducive to the application of immunotherapy. Our results may open up a new field for precision therapy.

There were still limitations in our study. We should state that the findings demonstrated in present research were obtained by bioinformatics analyzes and have not been verified by the required molecular biological assays. However, the investigation of this topic can be considered as another separate study, including our follow-up research plan.

## Figures and Tables

**Figure 1:** Screening of hypoxia-related genes. (a) Protein interactions among hypoxia-related genes. (b) Extracted 50 genes with the most connected nodes. (c) Univariate Cox regression analysis showed that 7 hypoxia-related genes were associated with the prognosis of patients. (d) 2 hypoxia-related genes were selected and multivariate Cox regression was used to establish the hypoxia risk model.

**Figure 2:** The predictive value of hypoxia risk score for the prognosis of oral squamous cell carcinoma. (a) Kaplan–Meier overall survival analysis of oral squamous cell carcinoma hypoxia high- and low-risk groups. (b) ROC curve shows the prognostic value of the patient's hypoxia risk score. (c) The mortality rate of patients in high- and low-risk groups. (d) Spearman correlation analysis of 2 hypoxia genes.

**Figure 3:** Prediction of patient risk in the hypoxia model. (a) Survival rates in the high- and low-risk patient groups. (b) Patient risk scores. (c) The expression levels of two hypoxia-related genes.

**Figure 4:** Analysis of immune cells in the high and low hypoxia risk groups. (a) The relative proportion of immune infiltration. (b) Differences in the level of immune cell infiltration between high- and low-risk groups.

**Figure 5:** (a) The expression difference of immune-related cells, ^*∗∗∗*^represents *p* < 0.001, ^*∗∗*^represents *p* < 0.01, ^*∗*^represents *p* < 0.05. (b–g) The expression levels of important family genes in high and low hypoxia risk groups.

**Figure 6:** GSEA enrichment in high hypoxia risk group.

**Figure 7:** GSEA enrichment in low hypoxia risk group.

## Data Availability

The datasets used and analyzed during the current study are available from the corresponding author upon reasonable request.
